The article "Sulfated Polysaccharides Derived from Hypnea valentiae and Their Potential of Antioxidant, Antimicrobial, and Anticoagulant Activities with In Silico Docking" was published in 2022. Journal: Evid Based Complement Alternat Med.

# Sulfated Polysaccharides Derived from *Hypnea valentiae* and Their Potential of Antioxidant, Antimicrobial, and Anticoagulant Activities with *In Silico* Docking

**DOI:** 10.1155/2022/3715806

**Published:** 2022-07-20

**Authors:** Kokila Palani, Balamuralikrishnan Balasubramanian, Arunkumar Malaisamy, Viji Maluventhen, Vijaya Anand Arumugam, Naif Abdullah Al-Dhabi, Mariadhas Valan Arasu, Karthika Pushparaj, Wen-Chao Liu, Maruthupandian Arumugam

**Affiliations:** ^1^Ethnopharmacology and Algal Biotechnology Division, Department of Botany, School of Life Sciences, Periyar University, Salem 636011, Tamil Nadu, India; ^2^Department of Food Science and Biotechnology, College of Life Science, Sejong University, Seoul 05006, Republic of Korea; ^3^Integrative Biology Division, International Centre for Genetic Engineering and Biotechnology (ICGEB), New Delhi, India; ^4^Department of Botany, Thiagarajar College, Madurai 625009, Tamil Nadu, India; ^5^Department of Human Genetics and Molecular Biology, Bharathiar University, Coimbatore 641046, Tamil Nadu, India; ^6^Department of Botany and Microbiology, College of Science, King Saud University, P.O. Box 2455, Riyadh 11451, Saudi Arabia; ^7^Department of Zoology, School of Biosciences, Avinashilingam Institute for Home Science and Higher Education for Women, Coimbatore, Tamil Nadu 641043, India; ^8^College of Coastal Agricultural Sciences, Guangdong Ocean University, Zhanjiang 524088, China

## Abstract

Carrageenan, a sulfated polysaccharide, was produced by certain species of marine red seaweeds, which have been used as a significant source of food, feed, and antibiotic agent throughout history due to their alleged human health benefits. The present study aimed to derive the polysaccharides from *Hypnea valentiae* and describe the biological applications. Carrageenan was characterized by FT-IR, C-NMR, AFM, and their antimicrobial, antioxidant, and anticoagulant capabilities; furthermore, the larvicidal effect of methanol extract was generated from the seaweed against *Aedes aegypti* larvae at various concentrations. The molecular docking experiments were carried out computationally for finding the molecular insight of the macromolecules and small molecules' interaction using GLIDE docking by using Schrodinger software. Antibacterial zones of inhibition in different concentrations are compared with the 40 mg/mL higher activity against bacterial pathogens. Carrageenan is strong in all antioxidant activities, with the overall antioxidant (70.1 ± 0.61%) of radical at 250 *μ*g/mL concentration being exhibited. The DPPH scavenging is effective in the inhibition of (65.74 ± 0.58%) radical at a concentration of 160 *μ*g/mL and the hydroxyl scavenging (65.72 ± 0.60%) of activity at a concentration of 125 *μ*g/mL being exhibited. Anticoagulant activities (APPT and PT) of carrageenan fraction were tested. *H. valentiae* and heparin sulphate shows higher activity of APTT (106.50 IU at 25 *μ*g/mL) in comparison with the PT test (57.86 IU at 25 *μ*g/mL) and the methanol extraction of higher larvicidal activity on *A. aegypti* (LC_50_ = 99.675 *μ*g/mL). In this study, the carrageenan was exploited through *in vitro* and *in silico* molecular docking studies against antimicrobial, antioxidant, and anticoagulant properties. The results were establishing the potentiality of the carrageenan which is an alternative source to control the mosquitocidal property in the future. Moreover, molecular docking of carrageenan against multiple targets results in −7 to −6 Kcal/mol binding score. Findings of carrageen from *in vitro* to *in silico* studies are needed for further validation of clinical pieces of evidence.

The article "Sulfated Polysaccharides Derived from Hypnea valentiae and Their Potential of Antioxidant, Antimicrobial, and Anticoagulant Activities with In Silico Docking" was published in 2022. Journal: Evid Based Complement Alternat Med.

## 1. Introduction

Marine macroorganisms are a rich source of functionally diversified bioactive compounds that play an active role in human nutrition and health. Seaweeds are a major source of sulfated polysaccharides, particles which are widely employed in food, feed, and medicine due to their rheological qualities as gelling and stabilizing agents [1, 2]. Sulfated polysaccharides have numerous biological and physiological activities, including antithrombotic [3], anticoagulant [4], antioxidant [5], antidiabetic [6], antibacterial [7], immunomodulatory [8, 9], antiviral [10], antiinflammatory [11], antinociceptive [12, 13], antitumor [14], and proinflammatory effects [15, 16]. Sulfated polysaccharides including agarans, galactans, and carrageenans are also available abundantly. Among these, carrageenan is a generic deviation of linear, sulfated galactans derived from species of red seaweeds [17]. Various investigations on the antioxidant and anticoagulant properties of seaweeds or their extracts have been published [18, 19]. Algal polysaccharides must be shown to serve a significant role as free-radical scavengers and antioxidants in the protection of oxidative damage in living organisms in current administration, and anticoagulants have long been used to treat blood during dialysis and surgery, as well as to treat disseminated intravascular coagulation and thrombosis in a variety of disorders and for *in vitro* blood testing [20, 21]. Mosquitoes, such as *Aedes aegypti,* are the deadliest since they act as a vector for a variety of diseases, including dengue fever, malaria, yellow fever, filariasis, and other types of chikungunya as well as Zika virus [22–25]. Furthermore, seaweed sulfated polysaccharide extracts contain primary and secondary metabolites including bioactive chemicals which are biodegradable into harmless products; it may be effective in mosquito larval control [26, 27].

The article "Sulfated Polysaccharides Derived from Hypnea valentiae and Their Potential of Antioxidant, Antimicrobial, and Anticoagulant Activities with In Silico Docking" was published in 2022. Journal: Evid Based Complement Alternat Med.

The standard new therapeutic approach is complicated, exhausting, expensive, time-consuming, and laborious. Computational methods such as molecular docking have played a critical role in rationalizing the road to drug discovery in order to overcome these obstacles. A molecular docking feature becomes a promising pharmaceutical research tool for screening candidates from drug libraries effectively [28]. In such studies, the ultimate goal was to find effective therapeutics for the carrageenan molecule extracted from marine algae. It is evaluated against antimicrobial, anticoagulant, and antioxidant activity using GLIDE docking in the maestro platform of Schrodinger software (Schrödinger Release 2021-2: Maestro, Schrödinger, LLC, New York, NY, 2021). Furthermore, the efficiency of the carrageenan compound was exploited with *in vitro* validation against the foresaid targets. Carrageenan is a sulfated polysaccharide, which is obtained by extraction from red seaweed species. It has been widely utilized in the food industry, agricultural, drug delivery, tissue engineering, and biosensor applications. Therefore, the present study investigated the isolation and biofunctional activities of carrageenan extracted from *H. valentiae,* characterization of structural properties using Fourier transform infrared (FT-IR) spectroscopy, ^13^C nuclear magnetic resonance (NMR), and atomic force microscopy (AFM) spectroscopy and evaluation of the biological properties such as antioxidant, antimicrobial, and anticoagulant activities with *in silico* molecular docking analysis.

## 2. Materials and Methods

### 2.1. Collection and Extraction of Sample

The red seaweed, *H. valentiae* (Turnur), was collected from Mandapam (Lat. 09°28′177N, Long. 79°18′536E) located on the southeast coastline of Ramanathapuram, Tamil Nadu, India. The seaweed specimen identification number was 1759. The sample was properly cleaned with seawater to remove all undesired pollutants such as sand particles and epiphytes and then thoroughly cleaned with tap water to discard all salt on the surface. The water was drained away, and the seaweed was laid out on the blotting paper to absorb any remaining moisture before being shade-dried at room temperature for 3 days and crushed into a fine powder. Following the completion of the sulfated polysaccharide extraction, the procedure was evaluated for 100 g of seaweed powder, which was soaked separately in acetone and methanol solvent in 7:3 for two days in a shaker at 200 rpm for 10 min. The process was repeated twice to ensure the dry biomass. This biomass was dried into a powder and dispersed in 1 L of 0.1 M HCL for 24 h with constant stirring at room temperature. The pellet was reextracted as above, and the supernatants were pooled. The supernatant was kept at 4°C overnight and precipitated with two volumes of absolute 1:1 and stirred continuously for 15 min, and then the precipitate was collected to separate carrageenan gel and distilled water. Carrageenan gel was then completely soaked in 96% alcohol for 1 h and stirred continuously. The carrageenan gel was separated from alcohol and distilled water by filtration. Subsequently, the mixture was centrifuged at 5000 rpm for 10 min, and the supernatant was neutralized with 1.0 M NaOH and poured in 100 mL of methanol. The carrageenan was freeze-dried by using a membrane at 70°C for a 24 h duration which was performed for further processing [29].

The article "Sulfated Polysaccharides Derived from Hypnea valentiae and Their Potential of Antioxidant, Antimicrobial, and Anticoagulant Activities with In Silico Docking" was published in 2022. Journal: Evid Based Complement Alternat Med.

### 2.2. Structural Analysis

Using an alpha FT-IR spectrophotometer and its technique, FT-IR was used to determine the functional groups of the carrageenan polysaccharides [30]. The characterization has been complemented by the ^13^C-NMR spectrum. The ^13^C-NMR spectrum of 10 mg of the carrageenan was dissolved in 0.5 mL solution in D_2_O which was recorded at 27°C on an NMR spectra Bruker model MHz 400 spectrometer. The proton chemical shift was expressed in parts per million (ppm). The substance was diluted in distilled water before being mixed with a solution of 200 *μ*g/mL carrageenan in 0.2 M NaOH. The carrageenan solutions were allowed to equilibrate for 1 h with NaOH prior to neutralization with HCl (pH∼6-7). Solutions were then passed through a 0.22 *μ*m filter and deposited onto 1 cm of a freshly cleaned glass plate surface (sample volume ∼60 *μ*L). Samples were dried for approximately 16 h in ambient conditions. Imaging of AFM was performed within 24 h of carrageenan deposition to avoid sample contamination.

### 2.3. Antibacterial Activity

Antibacterial studies were carried out on two Gram-positive bacteria (*Enterococcus faecalis* (MTCC 439) and *Staphylococcus aureus* (MTCC 96)) and Gram-negative bacteria (*Escherichia coli* (MTCC 443) and *Pseudomonas aeruginosa* (MTCC 741)). All the bacteria were obtained from the Research Laboratory, Microbiology Department, Periyar University, India. Positive control includes streptomycin. All bacterial cultures were incubated at 35°C for 24 h [31].

### 2.4. Antibiofilm Activity

To determine the effect of seaweed methanol extracts against antibiofilm activity, about 3.5 mL of nutrient broth and 1.5 mL of bacterial culture were added into sterile test tubes. 10 mg of sample was added to different concentrations of methanol extract (10, 20, 30, 40, and 50 *μ*g/mL) and additionally given into each tube. All tubes were incubated in a shaking incubator at 37°C for 24 h. After incubation, all tubes were washed with distilled water. All the tubes were breeze-dried for a few minutes and added 5 mL of crystal violet and then incubated at 37°C for 1 h. After incubation, we discarded the crystal violet from all the tubes and washed them with distilled water. About 5 mL of 95.0% ethanol was added into all test tubes and taken OD at 595 nm by UV-visible spectrophotometer [32], respectively. The antibiofilm activity was calculated using the formula of percentage:

(1) $$\begin{array}{c} \%\text{ of biofilm inhibition}=\frac{\text{control OD}-\text{treatment OD}}{\text{control OD}}\times 100. \end{array}$$

The article "Sulfated Polysaccharides Derived from Hypnea valentiae and Their Potential of Antioxidant, Antimicrobial, and Anticoagulant Activities with In Silico Docking" was published in 2022. Journal: Evid Based Complement Alternat Med.

### 2.5. Antioxidant Activity Measurement

#### 2.5.1. Total Antioxidant Property

The antioxidant activities of samples were evaluated by phosphomolybdenum complex formation according to the method [33]. About 0.5 mL sample extracts were added with 3 mL of reagent solution (0.6 M sulphuric acid, 28 mM sodium phosphate, and 4 mM ammonium molybdate). The test tubes were covered with foil and incubated in a water bath at 95°C for 90 min. After the samples had cooled to room temperature, the absorbance of the mixture was measured at 695 nm against the reagent blank. The reported results were mean values expressed as mg AAE/g sample.

### 2.6. Assay for Radical Scavenging In Vitro

#### 2.6.1. Scavenging Activity of DPPH (2,2-Diphenyl-1-picryl Hydrazyl)

Purified polysaccharides' DPPH-free radical-scavenging activity was assessed using Q-sepharose anion-exchange chromatography, as previously described by the technique [29, 34] with slight modifications. A solution of 3 mL of 0.1 mM methanolic solution DPPH was prepared. A respective blank sample of BHA and L-ascorbic acid was prepared by adding 100 *μ*g/mL. The discoloration of the sample was measured with a proper blank at 517 nm after incubation for 30 min at 30°C in the dark using a UV-Vis spectrophotometer. The samples' free radical scavenging activity was calculated using the following equation:

(2) $$\begin{array}{c} \%\text{ inhibition}=\left[\frac{\left(A1-A2\right)}{A1}\right]\times 100, \end{array}$$

where *A*1 is the absorption of the control and *A*2 is the absorption of the sample.

#### 2.6.2. Hydroxyl Radical Scavenging Assay

The capacity of the seaweed polysaccharides against the scavenging hydroxyl radical was evaluated using Fenton's reaction (Fe^2+^+H_2_O_2_⟶Fe^3+^+OH^−^+OH) according to the modification method described [35]. The extracts of methanol were evaporated in vials. The reaction mixture contained 1 mL of (EDTA) solution, 0.5 mL of EDTA (0.018%), and 1 mL of DMSO (0.85% v/v in 0.1 M phosphate buffer, pH 7.4), and 0.5 mL of ascorbic acid (0.22%) was added to each tube. The solution was incubated at 37°C for 15 min, and the presence of yellow color was measured spectrophotometrically at 510 nm against the blank sample. The mixture without the sample was treated as a control. The scavenging activity was calculated by the following equation:

(3) $$\begin{array}{c} \%\text{ inhibition}=\left\{1-\left[\frac{\left(A1\;-A2\right)}{A0}\right]\right\}\times 100, \end{array}$$

where *A*0 is the control, *A*1 is the absorption of the sample, and *A*2 is absorption without sodium salicylate.

The article "Sulfated Polysaccharides Derived from Hypnea valentiae and Their Potential of Antioxidant, Antimicrobial, and Anticoagulant Activities with In Silico Docking" was published in 2022. Journal: Evid Based Complement Alternat Med.

### 2.7. Anticoagulant Activity

#### 2.7.1. Activated Partial Thromboplastin Time (APTT)

For carrageenan fractions, APTT was calculated using a modified version of the methodology reported [36]. The positive and negative controls were heparin at a concentration of 5 g/mL and 0.9 percent w/v NaCl, respectively.

#### 2.7.2. Prothrombin Time (PT)

The methodology of [37] was also used to determine PT, with some modifications. The device was also programmed to perform the same procedure in APTT determination. Each poor-platelet plasma and carrageenan solution mixture was incubated for 3 min at 37°C. Then, 0.6 mL of prewarmed PT reagent was added, and the time for clot formation was also observed and repeated three times. For positive and negative control, heparin and NaCl were utilized, respectively.

### 2.8. Molecular Docking

Ligand preparation: for molecular docking studies, carrageenan structure was retrieved from the PubChem database (71597331) in a three-dimensional structure file (SDF) format, and furthermore, the structure was refined using the LigPrep module in Schrodinger's Maestro (v 12.8). The OPLS4 force field was applied, and 32 different states of stereoisomerism were derived (Schrödinger Release 2021-2: LigPrep, Schrödinger, LLC, New York, NY, 2021).

Protein preparation: we need to evaluate the antioxidant (2C0D & 5B6M), antimicrobial (1JIJ & 2XCT), and anticoagulant (5E8E) activity against sulfated polysaccharide computationally. The three-dimensional structure of proteins was retrieved from the database of Protein Data Bank (PDB). The X-ray crystallographic structures were imported into Maestro using the protein preparation wizard, and this module helps to solve the missing hydrogen bonds, create the disulfide bonds, and optimize (Schrödinger Release 2021-2: Protein Preparation Wizard; Epik, Schrödinger, LLC, New York, NY, 2021; Impact, Schrödinger, LLC, New York, NY; Prime, Schrödinger, LLC, New York, NY, 2021).

The article "Sulfated Polysaccharides Derived from Hypnea valentiae and Their Potential of Antioxidant, Antimicrobial, and Anticoagulant Activities with In Silico Docking" was published in 2022. Journal: Evid Based Complement Alternat Med.

The molecular docking was performed using the Glide package (ligand docking) in the Schrodinger suite. The standard precision docking method was applied and performed postdocking minimization and analyzed the results in pose viewer Schrödinger Release 2021-2: Glide, Schrödinger, LLC, New York, NY, 2021.

### 2.9. Mosquito Culture and Larvicidal Activity

*A. aegypti* mosquito larvae were collected from the Indian Council of Medical Research—Vector Control Research Centre, Madurai, Tamil Nadu, India. The mosquito larvae were fed a finely powdered mixture containing a 3 : 1 ratio of dog biscuits and Brewer's yeast for repeated generations at 25–30°C. According to the procedure used, adult mosquitoes were kept under standard environmental conditions as larvae [38]. Following this procedure, a mortality assay was carried out on fourth instar larvae [22, 39]. The test for the larvae effect of methanol extract derived from seaweed against mosquito larvae *A. aegypti* involved 10 mg of the sample in different concentrations for 50, 100, 200, and 500 *μ*L. Twenty larvae were added to 250 mL distilled water in triplicates, with 1 mL DMSO serving as a negative control H_2_O. Dead larvae were counted, and the proportion of dead larvae was estimated for the replicates after 24 and 48 h of exposure. Profit analysis was utilized to calculate average LC_50_ and LC_90_ (lethal concentration) values from the duplicates.

(4) $$\begin{array}{c} \%\text{ of mortality}=\frac{\text{number of dead larvae}}{\text{number of larvae introduced}}\times 100. \end{array}$$

### 2.10. Statistical Analysis

The results were examined using one-way analysis to calculate LC_50_, LC_90,_ and 95% fiducial limits of upper confidence and lower confidence of variance and standard values presented as the mean SD (ANOVA). The asterisk (^*∗*^, (^*∗∗*^, and ^*∗∗∗*^) denotes a significant difference from the control (*p* < 0.01, (*p* < 0.05, and *p* < 0.001).

## 3. Results

The FT-IR spectra of the carrageenan were isolated from the red seaweed *H. valentiae* and the absorption bands typical of carrageenan between the wave numbers 1000 and 3500 cm^−1^ clearly highlighted the functional groups in all of the analyzed samples (Figure 1, Table 1). The peaks at 3457.74 cm^−1^ correlate with O-H stretching H-bonding vibrations which indicated alcohols and phenols. The existence of alkanes was revealed by the similarity of the peaks found at 2349.36 cm^−1^. Furthermore, the peaks observed at 1687.22 cm^−1^ were attributed to alkenes. The aliphatic amines had an absorption peak position at 1187.22 cm^−1^ confirming the -C≡C- stretch. The spectral observations at 1222.18 cm^−1^ indicated asymmetric stretching of S-O, revealing the presence of sulfate [40]. The band at 1222.18–1030.72 cm^−1^ stretching of C-O was attributed to alcohols, carboxylic acids, esters, and ethers. C-H stretching vibrations indicated the existence of alkanes in the band between 1444.61 cm^−1^. The C-O-C of 3, 6-anhydro-L-galactose vibrations has been assigned to the peak at 920.72 cm^−1^. Aromatic group C-H stretching vibrations were as described to the peak 845.44 cm^−1^. The last peak which appears to be 650.30 cm^−1^ was related to -C≡C-H: C-H bending the presence of alkanes. The NMR spectra of the carrageenan provided more structural characterization, which is shown in Figure 2, respectively, and band assignment for a sample of *H. valentiae* polysaccharide. The NMR can be used to demonstrate the existence of different carrageenan units. The NMR spectrum was also a complex polymer signal from the anomeric proton at (78.30 ppm), and ring carbons (70.16 ppm) were assigned to 3,6-*α*-L-anhydrogalactose. The signal was assigned from the 75.02 ppm which was assigned to H-1 of *β*-D-galactose linked to *α*-L-galactose-6-sulfate. The signal at 102.86 ppm was attributed to carboxyl *β*-D-galactose.

The article "Sulfated Polysaccharides Derived from Hypnea valentiae and Their Potential of Antioxidant, Antimicrobial, and Anticoagulant Activities with In Silico Docking" was published in 2022. Journal: Evid Based Complement Alternat Med.

The surface topography of the carrageenan was studied with the help of AFM measurements in a contact mode. The AFM images of the carrageenan soft template and bright spot are shown in (Figure 3(a)). Moreover, the topography of the carrageenan can be observed with peaks and valleys distributed across the surface. Apart from this, huge numbers of deformed shapes with larger sizes can also be seen in the AFM image of the carrageenan (Figure 3(b)). The AFM is a significant source for detecting the morphology and size of the carrageenan macromolecules originating from 0.0 to 0.7 *μ*m. The carrageenan particles' average height which ranged from 0.00 to 0.72 *μ*m was also noted.

The antibacterial activity of the methanol extract was evaluated for the resistance to pathogenic bacteria which may cause infection in human beings. The methanol extract of *H. valentiae* inhibitory activity against *E*. *faecalis, S. aureus*, *E. coli,* and *P. aeruginosa* was identified. The pathogenic bacterial zone of inhibition in various concentrations of the methanol extract was compared to the 40 mg/mL higher inhibitory activity against four bacterial pathogens obtained in the results shown in (Figure 4) and Table 2, respectively. The antibacterial potential of methanol extracts depends upon the ability of permeation to the bacterial cell through the cell wall of bacteria. Moreover, the methanol extract had a minimum inhibitory bacterial effect against the Gram +ve strain rather than the Gram −ve strain. Therefore, the present study focused that both extracts demonstrated high significant antibacterial inhibition activity against Gram-negative bacteria rather than Gram-positive bacteria.

The article "Sulfated Polysaccharides Derived from Hypnea valentiae and Their Potential of Antioxidant, Antimicrobial, and Anticoagulant Activities with In Silico Docking" was published in 2022. Journal: Evid Based Complement Alternat Med.

The antibiofilm activity of methanol extract of *H. valentiae* has been investigated with bacterial potential against stains based on *E. faecalis* Gram +ve and *P. aeruginosa* Gram −ve bacterial activity obtained in the results shown in Table 3, respectively. The different concentrations of methanol extract (10, 20, 30, 40, and 50 *μ*g/mL) were tested. The highest activity against antibiofilm activity (11.1 ± 0.885 at 50 *μ*g/mL) methanol extract was recorded for *E. faecalis*. In *P*. *aeruginosa,* the inhibition of the biofilm activity rate as 14.3 ± 0.979 at 50 *μ*g/mL concentration of methanol extract was found. The percentage of inhibition in *E. faecalis* activity effect methanol extract was significantly higher than that in *P. aeruginosa*. The current study investigates the antibiofilm activity of *H. valentiae* extracts bacterial activity against two different bacterial strains.

Total antioxidant activity was measured to evaluate the antioxidant capacity of sulfated polysaccharides from *H. valentiae* extracts. The carrageenan extract was shown to reduce the total antioxidant scavenging activity of radicals (70.1 ± 0.61%) at 250 *μ*g/mL concentration rather than at the other concentrations of 50–250 *μ*g/mL of the displayed activities. Based on the findings visualized (Table 4) and noticed, the carrageenan was found to have significantly higher total antioxidant activities as compared with L-ascorbic acid (87.22 ± 0.80%) and BHA (81.99 ± 0.75%). The antiradical assay was determined by measuring the absorbance of the inhibition of DPPH radicals. The seaweed extract of sulfated polysaccharide showed that higher inhibition activity of these radicals (65.74 ± 0.58%) values for DPPH scavenging at 160 *μ*g/mL concentration rather than at the other concentrations. According to the results shown in (Table 4), carrageenan has the potential for radical scavenging activity when compared to the compounds of L-ascorbic acid (82.05 ± 0.73%) and BHA (79.01 ± 0.70%) that demonstrated effective DPPH neutralizing activity.

The hydrogen radical scavenging assay was used to determine the inhibition of hydroxyl (OH) radical formation, and the results showed that the scavenging activity of sulfated polysaccharide was significant with increasing concentrations. The extract of carrageenan inhibited the hydrogen peroxide scavenging activity of the OH radical (65.72 ± 0.60%) at 125 *μ*g/mL concentration rather than at the other concentrations of 25–125 *μ*g/mL of the exhibited activities. Furthermore, as shown in Table 4, carrageenan exhibited significantly higher hydroxyl radical activities when compared to L-ascorbic acid (81.140.73%) and BHA (77.930.70%).

The article "Sulfated Polysaccharides Derived from Hypnea valentiae and Their Potential of Antioxidant, Antimicrobial, and Anticoagulant Activities with In Silico Docking" was published in 2022. Journal: Evid Based Complement Alternat Med.

The study of anticoagulant activity was analyzed by the APTT and PT assays which demonstrated that the anticoagulant mechanism of carrageenan inhibits plasma coagulation release during the regular phase of the coagulation process blood clotting time (Table 5). The anticoagulant activity of carrageenan was exhibited higher in APTT (106.50 IU at 25 *μ*g/mL) when compared with the PT test (57.86* *IU at 25 *μ*g/mL) indicating the pathway to inhibition.

The carrageenan molecule was subjected to small molecular (ligand) docking, the antioxidant targets chosen as mitochondrial 2-cys peroxiredoxin (2C0D) from *Plasmodium falciparum* and crystal structure of human peroxiredoxin 6 (5B6M). The docking score results of −7 Kcal/mol indicate strong affinity among the complex molecules, and the interaction diagrams of 3D and 2D are represented in Figure 5. The antimicrobial target protein chosen as *S. aureus* tyrosyl-t RNA synthetase (1JIJ) and *S. aureus* gyrase topoisomerase II (2XCT) against the small molecule showed a strong affinity in their complex molecule with the least binding score of −6.894 Kcal/mol and with their interactive sites represented (Figure 6). The phytochemical exploited against antioxidant activity using auto dock tool results in −3.3 to −6 Kcal/mol binding score with *in vitro* validation, wherein in our case, it was shown as −7 Kcal/mol using Glide docking, Schrodinger [41]. The anticoagulant target protein was chosen as the crystal structure of thrombin (5E8E) from humans against carrageenan, showing the amino acid interaction as SER546 forms a hydrogen bond with the NH- group, and PO4 forms a hydrogen bond with the O- group with a docking score of −6.639. The structure was illustrated with 2D and 3D interaction maps with a pocket binding site (Figure 7, Table 6). Carrageenan extracted from *H. valentiae* was found to have the highest larvicidal activity against *A. aegypti* (LC_50_ = 99.675 *μ*g/mL; LC_90_ = 491. 453 mg/L) shown (Figure 8, Table 7). The larvicidal activity of seaweeds to the larvae of *A. aegypti* was determined to the inhibition effect of seaweed mortality larvae. Seaweed is a natural product, and particularly, halogenated terpenes might be exploited for the improvement of new larvicidal compounds and its prototype insecticidal agents.

## 4. Discussion

The present study on methanol extract of *H. valentiae* was tested for yield, antioxidant, antimicrobial, anticoagulant with *in-silico* molecular docking, and larvicidal activity properties. The extract effect is an important parameter for the chemical compounds which have been used in the screening of bioactive substances from red seaweeds enriched with secondary metabolites and have potential antioxidant, antimicrobial, and anticoagulant activities [42]. The FT-IR spectrum is one of the most important tools for polysaccharides and their spectroscopic assignments of functional groups. The O-H stretching of alcohol and phenol vibration from the intramolecular hydrogen bond corresponded to the absorption peak position at 3457.74 cm^−1^ [43]. The absorption peaks at 2349. 36–1687.22 cm^−1^ is attributable to C-H stretch and -C≡C- stretch alkane functional groups, which probably confirmed the polymer-bound water which is a characteristic feature of red seaweed polysaccharides [44]. These absorption bands were described as enhancing the activation of molecular chain movements. Furthermore, the absorption peaks at 1222.18–1030.72 cm^−1^ correspond to assignments of functional groups. C-O stretches alcohols, carboxylic acids, esters, and ethers from lipid triglycerides and fatty acids [45]. The absorption peak position at 1444.61 cm^−1^ is attributable to C-H symmetric stretching alkanes. Another characteristic peak 920.72 cm^−1^ is attributable to C-O-C stretch 3,6-anhydro-L-galactose in the presence of high sulfated polysaccharides [42]. The absorption peak 650.30 cm^−1^ is attributed to -C≡C-H: C-H sulfate group alkynes. 1030.72 cm^−1^ corresponds to the high molecular weight skeleton of sulfated D-galactans and carrageenan bands found in *H. valentiae* [46]. These absorption bounds of oxygen, nitrogen, and biofunctional groups confirmed the presence of polyphenol compounds, polysaccharides, and protein, primary, and secondary metabolites.

The article "Sulfated Polysaccharides Derived from Hypnea valentiae and Their Potential of Antioxidant, Antimicrobial, and Anticoagulant Activities with In Silico Docking" was published in 2022. Journal: Evid Based Complement Alternat Med.

The NMR spectroscopy is one of the efficient techniques for determining the structural characters of seaweed polysaccharides [47]. Recently, the report has demonstrated that the NMR spectrum used in the presence of different carrageenan components was observed to indicate the conversion of 3,6-*α*-L-anhydrogalactose units into its alditol derivatives anomeric protons containing *μ* and *ν* carrageenan [48]. Previous studies illustrate the occurrence of *β*-D-galactospectroscopic functional group of sulphated polysaccharides in the sugar residues, which are in conform that the trisaccharide branches on bacterial polysaccharide [49, 50]. Collectively, the literature has reported that *Gracilaria caudata* analyzes the structural features of *β*-D-galactos linked to *α*-L- galactose-6-sulfate, and methyl or pyruvate molecules are substituted by carrageenan polysaccharide [47, 51]. These reports indicated that the *α*-glycosidic peaks in the carrageenan backbone were partially broken [52]. NMR spectroscopy is also useful for recognizing the conformations of polysaccharides.

The AFM is single molecular spectroscopic technology to detect the conformation of morphological structures of polysaccharides in AFM images which provides a perfect observation of molecular assembling. The AFM provides visualization of the different types of sulfated polysaccharides such as curdlan [53], xanthan [54], carrageenan [55], xyloglucan [56], pectin [57], arabinoxylan [58], and starch [59]. The previous literature has functionalized the AFM based on the purpose of many fundamental food systems of carrageenan polysaccharides [48]. Similar reports have identified the height range in the structure of the food particles [49]. Based on the findings, the fibrous height of carrageenan was topographically similar to sulfated polysaccharides derived from the red seaweed [44]. The majority of the results from AFM analysis have reviewed the macromolecules of functional food polymers [60]. Therefore, AFM is nanostructure characteristics of polysaccharides from different food products. The conformation of polymers to identify numerous environmental conditions controlled the temperature [61].

The potential antibacterial activity of carrageenan polysaccharides from *H. valentiae* derivatives was evaluated to affect microbial pathogens of (*E*. *faecalis* and *S*. *aureus* (Gram +ve) and *E*. *coli* and P. *aeruginosa* (Gram −ve) organisms. The antibacterial activity was revealed to be strong against biologically multidrug-resistant pathogens *S. aureus and E. faecalis* [52]. In addition, numerous reports have described the antibacterial potential using algae extracts' strong effect on various bacterial pathogens such as *E. coli, S. aureus, and E. faecalis*. These pathogenic bacterial activities to enhancing the biostimulants of medicinal properties valuable for enhancing the mint and basil antimicrobial activity against bacteria [62]. Previous reports have analyzed the antibacterial activity against bacteria *Spatoglossum asperum* biological and pharmaceutical useful for valuable drugs [50]. The antibacterial activities of highly potential biomedical applications such as drug delivery, wound healing, and tissue engineering. The antibacterial capabilities could improve rapid healing by making a barrier against microbial contamination [63].

In the present study, *H. valentiae* were tested for antibiofilm activity potential against pathogenic strains that the reports revealed the methanol extract inhibited biofilm formation. Based on the reports, we have identified the biofilm activity inhibition of *Sargassum wightii* and *Halimeda gracillis* seaweed activity against antimicrobial pathogens and antibiofilm activity against various clinically significant pathogenic microorganisms [64]. The previous literature reported that the biofilm activities could be applied in different medical treatments to the prevention of various biofilm-related infections [65]. The biofilm pathogens are eco-friendly to presently used metal-based antifouling agents [66]. Collectively, the results have indicated the significant antibiofilm potential of the *Ulva lactuca* microbiocidal effect of different microorganisms that lead to the formation of cariogenic biofilm against the environment. It has been useful to the need for clinical studies to completely enhance the antibiofilm and mechanical properties of the new product [67].

The article "Sulfated Polysaccharides Derived from Hypnea valentiae and Their Potential of Antioxidant, Antimicrobial, and Anticoagulant Activities with In Silico Docking" was published in 2022. Journal: Evid Based Complement Alternat Med.

The antioxidant potential of polysaccharides for various free radical scavenging ability of higher polyphenol and flavonoids content was extracted, and they could have excellent antioxidant activity [68]. The antioxidant activity having higher polyphenol content in soluble fraction is observed to precipitate. The highly effective of polyphenol and flavonoids compounds with their hydroxyl group for scavenging free radicals [64]. The antioxidant activity of polysaccharides could protect the human system from reactive oxygen species which affect such macromolecules as membrane lipids, proteins, and DNA and lead to many functional disorders of the human body. In the current study, phenolic content was higher in methanol extract from *H. valentiae* which were screened for total antioxidant activity at 250 *μ*g/ml concentration. The highest total antioxidant activity is present in the methanol precipitate from *H. valentiae* (70.1 ± 0.61%). Previous literature reports have indicated the highest total antioxidant activity in the fractionated polysaccharides from *Turbinaria conoides* (246.6 mg AscAE/g) *Gracilaria filiforms* (353.3 AscAE mg/g), and *Enteromorpha compressa* (326.6 mg AscAE/g) [27]. Similar results have reported the highest total antioxidant activity occurred in extract sulfated polysaccharides *Sargassum tenerrimum* (22.0 ± 06) [69]. Similarly, the study reported the total antioxidant activity in aqueous extract of *codium* sp which showed the activity of 85.53 ± 0.25% [70]. The results revealed that the polysaccharides conformed that the total antioxidant activity which was the highest inhibition in the methanol extract from the red seaweed. The potential antioxidant activity screened for DPPH radical scavenging was due to their hydrogen donating ability. The free radical scavenging activity indicated a higher value in methanol extract from *H*. *valentiae* (65.74 ± 0.58%). Based on the results, the highest scavenging ability was present in the ethanolic precipitate of *S. wightii* (78.3 ± 0.25%) [64]. The antioxidant activity of polysaccharides extracted from Undaria pinnatifida showed that the highest inhibition of hydrogen peroxide screening ability [71]. In our study, the occurrence of the sulfate group to activate the hydrogen atom of the anomeric carbon through the sulfate content to adsorb the antioxidant exhibited the scavenging ability of *Sargassum thunbergii* [72]. The same other results demonstrated that the sulfated polysaccharide effect on inhibiting the formation of these radicals was higher in the extract from *Laminaria japonica* [73].

The article "Sulfated Polysaccharides Derived from Hypnea valentiae and Their Potential of Antioxidant, Antimicrobial, and Anticoagulant Activities with In Silico Docking" was published in 2022. Journal: Evid Based Complement Alternat Med.

The results showed that the exhibited hydroxyl radical formations determine the scavenging activity of sulfated polysaccharides was significantly higher than the extract from *H. valentiae* (65.72 ± 0.60%). The hydroxyl radical result reveals the damage to the biomolecules including protein, deoxyribonucleic acid, and polyunsaturated fatty acids in the human cell membrane. These costs must lead to the expansion of various infections including cancer (*Undaria pinnatifida*) [71]. Previous literature reports have demonstrated that sulfate groups of algal polysaccharides are various kinds of biological activities as antioxidant activity in radicals scavenging (*Sargassum thunbergii*) [72]. These results indicate the antioxidant activity of sulfate content had a significant source of hydroxyl radical scavenging ability [20].

The present investigation continues to the methanol extract screening anticoagulant activity. Anticoagulant activity has evaluated the APTT and PT assay that showed higher inhibition of the coagulant in the soluble fraction. The APTT and PT assay demonstrate the anticoagulant mechanism of the carrageenan as blood coagulation. The methanol precipitate of *H. valentiae* inhibited higher APTT (106.50 IU at 25 *μ*g/mL) and PT (57.86 IU at 25 *μ*g/mL). The anticoagulant property of the carrageenan was assessed using human plasma from healthy donors. The results found in the APTT assay showed that the carrageenan had higher coagulation properties. The main source of the anticoagulant property of the carrageenan appears could be antithrombic activity [16]. The anticoagulant pathway indicated the potentiality of the sulfated polysaccharides in spreading the coagulation time that paves the technique for more possibility for their application in pharmaceutical industry for drugs [74]. The ray skin dermatan sulfated DS showed higher anticoagulant activity of the skin DS as shown by APTT and PT anticoagulant drug of interest potentially useful in therapy. The report suggested the higher content of the sulfate group which presented higher coagulant property [75].

The article "Sulfated Polysaccharides Derived from Hypnea valentiae and Their Potential of Antioxidant, Antimicrobial, and Anticoagulant Activities with In Silico Docking" was published in 2022. Journal: Evid Based Complement Alternat Med.

Sulfated polysaccharides are heterogeneous natural polymers found in massive quantities in marine algae with a wide range of therapeutic applications due to their chemical structure and composition. The identification of chemicals that reduce inflammation is of importance because inflammation plays a role in illnesses. Antiinflammation activity has been determined using a variety of approaches. With results of in vitro assays, several derivatives of carrageenan oligosaccharides had better antioxidant activity than carrageenan oligosaccharides, indicating that chemical modification of carrageenan oligosaccharides could improve their antioxidant activity [76]. The investigations of these studies showed noticeable significance, and the resultant complex molecules amino acid interaction with bond length are depicted in Table 7. Carrageenan had been exploited with antimicrobial, antiviral, and anticancer activity. The current research observed a significant interaction of the carrageenan with multiple targets resulting majorly around −7 to −6 Kcal/mol binding score [28, 77].

The mosquito larvicidal activity of methanol extract from *H. valentiae* has been found in the highest larvicidal activity than the control *A. aegypti* (LC_50_ = 99.675 *μ*g/mL; LC_90_ = 491.453 mg/L). The present investigation focused on the larvicidal efficacy of the potential effect on the development of *H. valentiae* against *A. aegypti*. Based on the results observed in *Padina australis* (LC_50_ = 82.55 mg/mL), *Sargassum binderi* (LC_50_ = 160.07) mg/mL, *Bryopsis pennata* (LC_50_ = 192.43 mg/mL), the methanol extract was much effective on *A. aegypti* larvicidal activities. The report provided information on numerous effects using different seaweed extracts of *A. aegypti* [78]. *Gracilaria filiforms* has been reviewed in the literature larvicidal activity against the larvae *Anopheles stephensi* in which the higher inhibition is LC_50_ = 0.255867 and LC_90_ = 3.434589 mg/L [27]. The mosquito activity of the current research reported damage and shrinkage of cells from the midgut epithelium of the seaweed treated larvae *Anopheles stephensi* and *A. aegypti* which is (LC_50_: 58.34; LC_90_: 114.91). The application of the seaweed extracts is derived from terrestrial aromatic and medicinal values [64]. *Halimeda macroloba* has been reported in the literature in the past (LC_50_—1119.0; LC_90_—1890.3) and similarly *Ulva lactuca* (LC_50_—952.9; LC_90_—1830.4) and *Caulerpa racemosa* (LC_50_—886.0; LC_90_—1790.1) [79]. The same was reported to show the activity against the larvicidal activity of *Hypnea muciformis* and *Padina gymnospora* [80]. Based on the results responsible for the larvicidal action, demonstrating the use of seaweed extracts has high potential as a mosquito control strategy.

The article "Sulfated Polysaccharides Derived from Hypnea valentiae and Their Potential of Antioxidant, Antimicrobial, and Anticoagulant Activities with In Silico Docking" was published in 2022. Journal: Evid Based Complement Alternat Med.

## 5. Conclusion

The findings of this study suggested that the natural carrageenan derivatives with high sulfate content have greater radical scavenging antioxidant and antibacterial properties. Carrageenan from red seaweeds has also been shown to have *in vitro* anticoagulant functions, confirming its explicit role in the coagulation pathway. However, more research is needed to confirm that seaweeds have high mosquitocidal activity in the future. In addition, the carrageenan was evaluated computationally using glide ligand—molecular docking with multiple targets of antimicrobial, antioxidant, and anticoagulant activity. The minimal binding score explicits the strong affinity among the complex molecules. However, our potential candidate needs to further validate the *in vivo* model and extend it to clinical trials.

## Figures and Tables

**Figure 1:** FT-IR spectrum of the carrageenan from *Hypnea valentiae.*

**Figure 2:** ^13^C-NMR spectrum of the carrageenan from *Hypnea valentiae.*

**Figure 3:** AFM of the carrageenan from *Hypnea valentiae.*

**Figure 4:** The zone of inhibition for methanol extracts of *Hypnea valentiae* activity against (a) *E. coli*, (b) *E. faecalis*, (c) *P. aeruginosa*, and (d) *S. aureus.* 1—methanol, 2—antibiotic s*treptomycin*, 3—methanol extract 10 mg/mL, 4—methanol extract 20 mg/mL, and 5—methanol extract 40 mg/mL.

**Figure 5:** Molecular docking of the carrageenan against antioxidant targets (i) 2COD protein. (a) 3D surface mess map interaction site. (b) 3D complex interaction. (c) 2D complex interaction. (ii) 5B6M. (d) 3D surface mess map interaction site. (e) 3D complex interaction. (f) 2D complex interaction.

**Figure 6:** *Staphylococcus aureus* tyrosyl-tRNA synthetase docked with carrageenan. (a) 3D surface mess map interaction site. (b) 3D interaction site. (c) 2D interaction map. *S. aureus* gyrase topoisomerase II docked with carrageenan. (d) 3D surface mess map interaction site. (e) 3D interaction site. (f) 2D interaction map.

**Figure 7:** Molecular docking of the carrageenan against anticoagulant target proteins of 5EBE. (a) pocket 3D interaction site. (b) 3D complex interaction. (c) 2D complex interaction.

**Figure 8:** Larvicidal activity of *Hypnea valentiae*.

**Table 1:** Interpretation of functional groups in the carrageenan using FT-IR.

Peak position (wave number cm^−1^)	Spectroscopic assignments	Functional groups
3457.74 cm^−1^	O-H stretch, H-bonding	Alcohol, phenol
2349.36 cm^−1^	C-H stretch	Alkanes
1687.22 cm^−1^	-C≡C- stretch	Alkenes
1187.22 cm^−1^	C-N stretch	Aliphatic amines
1222.18-1030.72	C-O stretch	Alcohols, carboxylic acids, esters, and ethers
1444.61 cm^−1^	C-H bend	Alkanes
920.72 cm^−1^	C-O-C stretch	3, 6-anhydro-L-galactose
845.44 cm^−1^	C-H stretch	Aromatics
650.30 cm^−1^	-C≡C-H : C-H bend	Alkynes

The article "Sulfated Polysaccharides Derived from Hypnea valentiae and Their Potential of Antioxidant, Antimicrobial, and Anticoagulant Activities with In Silico Docking" was published in 2022. Journal: Evid Based Complement Alternat Med.

**Table 2:** The zone of inhibition for methanol extracts of *Hypnea valentiae* activity against bacterial species.

Bacteria	Zone of inhibition (mm)				
	**1**	**2**	**3**	**4**	**5**
*E. coli*	3.0 ± 0.577	5.0 ± 0.577	0	1.0 ± 0.577	1.0 ± 0.274
*E. faecalis*	1.0 ± 0.577	9.0 ± 1.155	0.00	1.0 ± 0.288	2.0 ± 0.577
*P. aeruginosa*	2.0 ± 0.320	0.0 ± 0.000	0.00	3.0 ± 0.111	5.0 ± 0.412
*S. aureus*	1.0 ± 0.000	8.0 ± 1.155	0	0.0 ± 0.000	0.0 ± 0.000

^*∗*^Data are mean=SE (*n*-3). 1—methanol, 2—antibiotic S*treptomycin*, 3—methanol extract 10 mg/mL,4—methanol extract 20 mg/mL, and 5—methanol extract 40 mg/mL.

**Table 3:** The effect of *Hypnea valentiae* methanol extracts on antibiofilm activity *E. faecalis* and *P. aeruginosa.*

Pathogens	Concentrations of methanol extracts of *H. valentiae* (*μ*g/mL)				
	**10**	**20**	**30**	**40**	**50**
*E. faecalis*	1.0 ± 0.211	4.2 ± 0.392	7.5 ± 0.555	10.0 ± 0.709	11.1 ± 0.885
*P. aeruginosa*	4.0 ± 0.380	7.0 ± 0.885	9.1 ± 0.692	12.0 ± 0.883	14.3 ± 0.979

^*∗*^Data are mean=SE (*n*-3).

**Table 4:** Antioxidant activity of *Hypnea valentiae* methanol extract.

Extract/positive control	Antioxidant activity, %		
	DPPH, *μ*g/mL	OH, *μ*g/mL	Total antioxidant, *μ*g/mL
Carrageenan	65.74 ± 0.58	65.72 ± 0.60	70.1 ± 0.61
BHA	79.01 ± 0.70	77.93 ± 0.70	81.99 ± 0.75
L-ascorbic acid	82.05 ± 0.73	81.14 ± 0.73	87.22 ± 0.80

**Table 5:** Anticoagulant activity of *Hypnea valentiae.*

Extraction/control	Clotting time	
	APTT, 25 *μ*g/mL	PT, 25 *μ*g/mL
Carrageenan	106.4 ± 0.65	57.3 ± 0.70
Heparin-sulfate	175.2 ± 0.85	126.5 ± 0.88

**Table 6:** Molecular docking of the carrageenan molecule against three different activities of 5 multiple targets, the bond length in which the range below 3 Å is hydrogen bond interaction.

S No	PDB	Target activity	Amino acid interaction site	Bond length, Å	Docking score
1	2C0D	Antioxidant	GLY164, ASN166, ASN165	2.22, (2.07, 2.67), 2.50	−7.465
2	5B6M	Antioxidant	VAL189, PHE207, LYS204, VAL187, PHE202	(2.54, 2.25), (2.32, 2.25), 2.13, 1.97, (2.58, 2.45)	−6.227
3	5E8E	Anticoagulant	ASN415, SER546, TRP370	2.38, 2.28, (2.42, 2.39)	−6.639
4	1JIJ	Antimicrobial	GLN196, ASP40, LYS84, ASP195	2.53, 1.95, (1.66 and 2.38) and 1.82	−6.894
5	2XCT	Antimicrobial	GLU1456, LYS1375, SER1453	(1.60, 2.01), (1.78, 2.21) and (2.34, 2.10)	−4.363

The article "Sulfated Polysaccharides Derived from Hypnea valentiae and Their Potential of Antioxidant, Antimicrobial, and Anticoagulant Activities with In Silico Docking" was published in 2022. Journal: Evid Based Complement Alternat Med.

**Table 7:** The effect of aqueous and methanol extract of the *Hypnea valentiae* against *Aedes aegypti* larvae.

Mosquito species	Extract	Hours	LC_50_ (*μ*g/mL)	95% confidence limit		LC_90_ (*μ*g/mL)	95% confidence limit		*x* ^2^	df
				Lower	Upper		Lower	Upper		
*Aedes aegypti*	Control (H_2_O)	24	316.083	236.821	488.167	2322.664	1171.696	8645.237	2.823	10
		48	289.440	208.435	486.467	3219.817	1359.596	20753.085	2.514	10
	Methanol (40 *μ*g/250 mL)	24	171.464	134.073	224.234	1081.894	657.746	2603.426	3.415	10
		48	99.675	76.920	123.824	491.453	345.703	876.642	6.845	10

## Data Availability

The data presented in this study are available on request from the corresponding authors.
